# Systematic Analysis of CXC Chemokine–Vascular Endothelial Growth Factor A Network in Colonic Adenocarcinoma from the Perspective of Angiogenesis

**DOI:** 10.1155/2022/5137301

**Published:** 2022-10-04

**Authors:** Yongli Situ, Xiaoyong Lu, Yongshi Cui, Qinying Xu, Li Deng, Hao Lin, Zheng Shao, Jv Chen

**Affiliations:** ^1^Department of Parasitology, Guangdong Medical University, Zhanjiang, 524023 Guangdong, China; ^2^Orthopedic Center, Affiliated Hospital of Guangdong Medical University, Zhanjiang, 524023 Guangdong, China; ^3^Department of Pharmacy, Affiliated Hospital of Guangdong Medical University, Zhanjiang, 524001 Guangdong, China

## Abstract

**Background:**

Tumor angiogenesis plays a vital role in tumorigenesis, proliferation, and metastasis. Recently, vascular endothelial growth factor A (*VEGFA*) and CXC chemokines have been shown to play vital roles in angiogenesis. Exploring the expression level, gene regulatory network, prognostic value, and target prediction of the CXC chemokine-VEGFA network in colon adenocarcinoma (COAD) is crucial from the perspective of tumor angiogenesis.

**Methods:**

In this study, we analyzed gene expression and regulation, prognostic value, target prediction, and immune infiltrates related to the CXC chemokine-VEGFA network in patients with COAD using multiple databases (cBioPortal, UALCAN, Human Protein Atlas, GeneMANIA, GEPIA, TIMER (version 2.0), TRRUST (version 2), LinkedOmics, and Metascape).

**Results:**

Our results showed that *CXCL1/2/3/5/6/8/11/16/17* and *VEGFA* were markedly overexpressed, while *CXCL12/13/14* were underexpressed in patients with COAD. Moreover, genetic alterations in the CXC chemokine-VEGFA network found at varying rates in patients with COAD were as follows: *CXCL1/2/17* (2.1%), *CXCL3/16* (2.6%), *CXCL5/14* (2.4%), *CXCL6* (3%), *CXCL8* (0.8%), *CXCL11/13* (1.9%), *CXCL12* (0.6%), and *VEGFA* (1.3%). Promoter methylation of *CXCL1/2/3/11/13/17* was considerably lower in patients with COAD, whereas methylation of *CXCL5/6/12/14* and *VEGFA* was considerably higher. Furthermore, *CXCL9/10/11* and *VEGFA* expression was notably correlated with the pathological stages of COAD. In addition, patients with COAD with high *CXCL8/11/14* or low *VEGFA* expression levels survived longer than patients with dissimilar expression levels. CXC chemokines and *VEGFA* form a complex regulatory network through coexpression, colocalization, and genetic interactions. Moreover, many transcription factor targets of the CXC chemokine-VEGFA network in patients with COAD were identified: RELA, NFKB1, ZFP36, XBP1, HDAC2, SP1, ATF4, EP300, BRCA1, ESR1, HIF1A, EGR1, STAT3, and JUN. We further identified the top three miRNAs involved in regulating each CXC chemokine within the network: miR-518C, miR-369-3P, and miR-448 regulated *CXCL1*; miR-518C, miR-218, and miR-493 regulated *CXCL2*; miR-448, miR-369-3P, and miR-221 regulated *CXCL3*; miR-423 regulated *CXCL13*; miR-378, miR-381, and miR-210 regulated *CXCL14*; miR-369-3P, miR-382, and miR-208 regulated *CXCL17*; miR-486 and miR-199A regulated *VEGFA*. Furthermore, the CXC chemokine-VEGFA network in patients with COAD was notably associated with immune infiltration.

**Conclusions:**

This study revealed that the CXC chemokine-VEGFA network might act as a prognostic biomarker for patients with COAD. Moreover, our study provides new therapeutic targets for COAD, serving as a reference for further research in the future.

## 1. Background

Colon cancer is a common malignant tumor of the digestive tract. The incidence and mortality of colon adenocarcinoma (COAD) are the third highest of all cancer types [1]. Since the early diagnosis of COAD remains difficult, its mortality is increasing yearly [2]. Approximately 50% of COAD patients relapse or die within five years [3]. Although using bioactive materials in anticancer drugs improves their overall therapeutic effects [4, 5], finding new biomarkers and therapeutic targets for early diagnosis remains the most critical initial step in the prevention and treatment of COAD.

Chemokines are a family of small heparin-binding proteins 8–10 kDa in size. Four subgroups exist within the chemokine family (CXC, CC, CX3C, and C). The CXC subgroup has been shown to play a crucial role in angiogenesis in physiological and pathological settings [6]. Recently, the role of CXCL in regulating tumor angiogenesis has attracted increasing interest [7]. Different members of the CXC chemokines subgroup can promote or inhibit angiogenesis, thus promoting or inhibiting tumor growth [8]. Multiple factors have been identified as regulators of angiogenesis. However, CXC chemokines are a unique family of cytokines that regulate angiogenesis in several ways [9]. Vascular endothelial growth factor A (*VEGFA*) is a vital factor that plays an essential role in tumor angiogenesis and development [10]. Sunitinib, a *VEGFA* inhibitor, has been used to treat advanced renal cell carcinoma. However, the side effects of sunitinib can be quite severe and include kidney and cardiovascular damage [11]. CXC chemokines and *VEGFA* are heavily regulated during tumor angiogenesis. *CXCL12* can promote a malignant phenotype by promoting the clonal growth of colorectal cancer cells and regulating the expression of *VEGF* and *ICAM-1* [12].

Multiple online databases were used to explore the expression level, gene regulation network, prognostic value, and regulation targets of the CXC chemokine-VEGFA network in patients with COAD from an angiogenic perspective in this study. In addition, we aimed to identify the relationship between CXC chemokine and *VEGFA* expression and the development and prognosis of COAD, as well as to provide new insights into targeted therapies for patients with COAD.

## 2. Methods

### 2.1. UALCAN Analysis

UALCAN (http://ualcan.path.uab.edu/analysis.html) is a free online database that provides analysis based on The Cancer Genome Atlas (TCGA) and MET500 cohort data [13]. The “Expression Analysis” module from the UALCAN database was utilized to examine TCGA gene expression data, and the following screening criteria were applied: (1) gene: CXC chemokines and *VEGFA*, (2) dataset: COAD, and (3) threshold setting conditions: *P* value cutoff = 0.05. A Student's *t*-test was used for the comparative analysis [14–16]. Data were obtained on February 14, 2022.

### 2.2. Human Protein Atlas Analysis

The Human Protein Atlas (https://www.proteinatlas.org/), an open-access resource, provides analyses of specific human genes and proteins [17]. Screening condition: (1) gene: CXC chemokines and *VEGFA*, (2) section: tissue and pathology, (3) tissue: colon and COAD, and (4) picture of tissue types: normal colon tissue and COAD. Data were obtained on February 14, 2022.

### 2.3. GEPIA

GEPIA (http://gepia.cancer-pku.cn/index.html) is an analysis tool that delivers RNA sequencing expression data from 9,736 cancerous and 8,587 noncancerous samples [18]. Gene (CXC chemokines and *VEGFA*), dataset (COAD), and threshold conditions (*P* value cutoff = 0.05) were set as screening criteria. The expression of CXC chemokines and *VEGFA*, as well as the pathological stage of COAD, was analyzed using a Student's *t*-test. The prognosis of patients with COAD was analyzed using the Kaplan–Meier curve [14–16]. Data were obtained on February 15, 2022.

### 2.4. cBioPortal Analysis

cBioPortal (http://cbioportal.org) is a free online database for visualizing, studying, and analyzing cancer genomic data [19]. The analysis of genetic alterations in the CXC chemokine-VEGFA network was conducted using cBioPortal in this study. Overall, 636 samples of COAD were analyzed. A *z*-score threshold of ±2.0 was used to calculate mRNA expression *z*-scores for all samples (log RNA Seq V2 RSEM). CXC chemokines and *VEGFA* were the chosen genes [14–16]. Data were obtained on February 15, 2022.

### 2.5. STRING Analysis

STRING (https://string-db.org/cgi/input.pl) is a free online database that helps researchers analyze all publicly available sources of protein–protein interaction (PPI) data [20]. We created the PPI network interaction using STRING in this study. The screening criteria were set as follows: (1) confidence: 0.400 and (2) species: *Homo sapiens* [14, 15]. Data were obtained on February 16, 2022.

### 2.6. GeneMANIA Analysis

GeneMANIA (http://www.genemania.org) is a free online database that creates PPI networks and analyzes gene function [21]. The interaction networks were built using this database to explore the roles of CXC chemokines and *VEGFA* [14–16]. Data were obtained on February 16, 2022.

### 2.7. Metascape Analysis

Metascape (https://metascape.org) is a free online gene function analysis tool that assists users in using current common bioinformatics analysis approaches to batch gene and protein analysis to predict function [22]. We conducted Gene Ontology (GO) function and Kyoto Encyclopedia of Genes and Genomes (KEGG) pathway enrichment analyses of the CXC chemokine-VEGFA network in COAD using Metascape [14–16]. Data were obtained on February 17, 2022.

### 2.8. TRRUST Analysis

TRRUST (https://www.grnpedia.org/trrust/) is a free online database for human transcriptional regulatory networks [23]. We sought to discover critical factors regulating the expression of the CXC chemokine-VEGFA network in COAD patients using TRRUST. The “Find key regulators for query genes” module of TRRUST, species (human), and gene (CXC chemokines and *VEGFA*) were chosen in this study [14–16]. Data were obtained on February 17, 2022.

### 2.9. LinkedOmics Analysis

LinkedOmics (http://www.linkedomics.org/) is a free database that provides methods for analyzing and comparing cancer multiomics data [24]. The “LinkInterpreter” module of LinkedOmics was used to derive biological insights into miRNA target enrichment and transcription factor target enrichment of the CXC chemokine-VEGFA network. A minimum number of three genes (size), cancer type (COAD), a simulation of 500, gene (CXC chemokines and *VEGFA*), and target dataset (RNA-seq) were chosen in this study [14–16]. Data were obtained on February 18, 2022.

### 2.10. TIMER Analysis

TIMER (https://cistrome.shinyapps.io/timer/) is a free online platform for systematically analyzing tumor-infiltrating immune cells [25]. The “Gene module” of TIMER was used to assess the correlation between the expression level of the CXC chemokine-VEGFA network and tumor-infiltrating immune cells [14–16]. Data were obtained on February 18, 2022.

## 3. Results

### 3.1. Aberrant Expression of CXC Chemokine-VEGFA Network

The expression levels of the CXC chemokine-VEGFA network in patients with COAD compared with those without COAD were analyzed. We observed that the transcriptional levels of *CXCL1/2/3/5/6/8/11/16/17* and *VEGFA* were remarkably upregulated in (1) sex (male and female), (2) pathological stage (stage 1–4), and (3) sample type (COAD) (*P* < 0.05) (Figures 1(a1)–1(g3) and 1(k1)–1(m3)). However, *CXCL12/13* expression level in patients with COAD was downregulated in (1) sex (male and female), (2) pathological stage (stage 1–4), and (3) sample type (COAD) (*P* < 0.05) (Figures 1(h1)–1(i3)). *CXCL14* expression level in patients with COAD was downregulated in (1) sex (male), (2) pathological stage (stage 2), and (3) sample type (COAD) (*P* < 0.05) (Figures 1(j1)–1(j3)). In addition, immunohistochemical results validated the differential expression of the CXC chemokine-VEGFA network between patients with COAD and those without COAD (Figure 2). The pathological stage of COAD and the differential expression of the CXC chemokine-VEGFA network were assessed in this study. The pathological stage in patients with COAD and the expression of *CXCL9/10/11* and *VEGFA* were found to have a significant correlation (*P* < 0.05) (Figure 3). Subsequently, the prognostic ability of the CXC chemokine-VEGFA network expression in COAD patients was evaluated. The overall survival was longer in COAD patients when levels of *CXCL8/11/14* expression were higher (*P* ≤ 0.05) (Figures 4(a)–4(c)) or when levels of VEGFA expression were lower (*P* < 0.05) (Figure 4(d)).

### 3.2. Promoter Methylation and Genetic Alteration Analyses of CXC Chemokine-VEGFA Network

TCGA was utilized to analyze the genetic alterations of the CXC chemokine-VEGFA network in patients with COAD. As a result, the expression of *VEGFA* was altered by 1.3% in COAD patients (Figure 5). COAD patients had higher promoter methylation levels of *VEGFA* than individuals without COAD (Figure 6). However, differences in chemokine expression levels in patients with COAD, *CXC1/2/17* (2.1%), *CXCL3/16* (2.6%), *CXCL5/14* (2.4%), *CXCL6* (3%), *CXCL8* (0.8%), *CXCL11/13* (1.9%), and *CXCL12* (0.6%), were found (Figure 5). Similarly, the promoter methylation level of *VEGFA* and *CXCL5/6/12/14* was higher in COAD patients than in healthy individuals (Figure 6). Conversely, healthy individuals had higher promoter methylation levels of *CXCL1/2/3/11/13/17* expression than patients with COAD (Figure 6).

### 3.3. CXC Chemokines and *VEGFA* Interaction Network

The potential interactions between CXC chemokines and *VEGFA* in patients with COAD were explored. Overall, 13 nodes and 68 edges were obtained in the PPI network using STRING software (Figure 7(a)). The average node degree and local clustering coefficient of the PPI network were 10.5 and 0.908, respectively. Furthermore, the CXC chemokine-VEGFA network (33 genes and 2,152 edges) was linked to a complex interaction network through shared protein domains, coexpression, predicted, colocalization, and genetic interactions using GeneMANIA (Figure 7(b)). Moreover, cell chemotaxis, chemokine and cytokine receptor binding, chemokine and cytokine activity, leukocyte chemotaxis, and migration were the major functions of the CXC chemokine-VEGFA network in COAD patients (Figure 7(b)). In brief, CXC chemokines were connected to and interacted with *VEGFA* in a complex network.

### 3.4. GO and KEGG Pathway Enrichment Analyses

Metascape was utilized to analyze the functions of the CXC chemokine-VEGFA network in patients with COAD. We found that the biological processes connected with CXC chemokines and *VEGFA* were mainly related to leukocyte chemotaxis, myeloid leukocyte migration, positive regulation of leukocyte chemotaxis, lymphocyte migration, and regulation of multiorganism processes (Figure 8(a)). Moreover, chemokine and cytokine activity, heparin binding, and growth factor activity were the main molecular functions of CXC chemokine-VEGFA network expression (Figure 8(b)). The KEGG pathway of the CXC chemokine-VEGFA network in COAD was mainly involved in cytokine-cytokine receptor interaction, rheumatoid arthritis, interleukin- (IL-) 17 signaling pathway, and nuclear factor kappa B (NF-*κ*B) signaling pathway (Figure 8(c)).

### 3.5. Transcription Factor Targets Involved with the CXC Chemokine-VEGFA Network

Potential transcription factors involved with the CXC chemokine-VEGFA network in COAD patients were identified (Table 1). v-rel reticuloendotheliosis viral oncogene homolog A (RELA) and nuclear factor-kappa light polypeptide gene enhancer in B cells 1 (NFKB1) were the critical transcription factors involved with *CXCL1/2/5/8/12* and *VEGFA* in COAD patients (*P* < 0.001). In addition, *CXCL8* and *VEGFA* were found to be regulated by ZFP36 ring finger protein (ZFP36), X-box-binding protein 1 (XBP1), histone deacetylase 2 (HDAC2), activating transcription factor 4 (ATF4), E1A-binding protein p300 (EP300), early growth response 1 (EGR1), signal transducer and activator of transcription 3 (STAT3), and Jun proto-oncogene (JUN) (*P* < 0.01). Furthermore, *CXCL1/5/14* and *VEGFA* were found to be regulated by Sp1 transcription factor (SP1) (*P* < 0.001). Breast cancer 1 (BRCA1) was the key transcription factor involved with *CXCL1* and *VEGFA* in COAD patients (*P* < 0.01). Finally, estrogen receptor 1 (ESR1) and hypoxia-inducible factor 1 alpha subunit (HIF1A) regulated the functions of *CXCL12* and *VEGFA* (*P* < 0.01).

### 3.6. miRNA Targets of CXC Chemokine-VEGFA Network

The top three miRNA targets of the CXC chemokine-VEGFA network were obtained (Table 2). The miRNA targets of *CXCL1* were miR-518C, miR-369-3P, and miR-44. In addition, miR-518C, miR-218, and miR-493 were identified as potential miRNA targets that regulate *CXCL2*. Furthermore, we observed that *CXCL3* was regulated by miR-448, miR-369-3P, and miR-221. miRNA target of *CXCL13* is miR-423. Moreover, miR-378, miR-381, and miR-210 were identified as potential miRNA targets that regulate *CXCL14*. *CXCL17* is regulated by miR-369-3P, miR-382, and miR-208. Furthermore, our results showed that miR-486 and miR-199A are potential miRNA targets that regulate *VEGFA*.

### 3.7. Correlation of CXC Chemokine-VEGFA Network Expression and Differentially Expressed Genes

mRNA sequencing data of 379 patients with COAD were obtained from TCGA database of LinkedOmics. Upon analysis, 19,828 genes were closely related to *CXCL1/2/3/5/6/8/11/12/13/14/16/17* and *VEGFA* (Figure 9). Among these, we observed that 11,701 and 8,127 genes were negatively and positively correlated with *CXCL1* expression, respectively (Figure 9(a1)). Moreover, 50 genes had a notable positive or negative correlation with *CXCL1* expression in COAD patients (*P* < 0.05) (Figures 9(a2) and 9(a3)). *CXCL1* expression was strongly associated with the increased expression of *CXCL3* (Pearson's correlation coefficient (PCO) = 0.8921, *P* = 4.226*e*–132) (Figure 10(a1)), *CXCL2* (PCO = 0.8121, *P* = 3.304*e*–90) (Figure 10(a2)), and *ZC3H12A* (Pearson's correlation = 0.6531, *P* = 1.882*e*–47) (Figure 10(a3)).

Furthermore, we found that 11,137 and 8,691 genes were negatively and positively correlated with *CXCL2* expression, respectively (Figure 9(b1)). Among them, 50 genes had a marked positive or negative correlation with *CXCL2* expression in COAD patients (Figures 9(b2) and 9(b3)). Moreover, the expression of *CXCL2* was positively associated with the expression of *CXCL3* (PCO = 0.8728, *P* = 1.601*e*–119) (Figure 10(b1)), *CXCL1* (Pearson's correlation = 0.8121, *P* = 3.304*e*–90) (Figure 10(b2)), and *ZC3H12A* (PCO = 0.6447, *P* = 6.735*e*–46) (Figure 10(b3)). Furthermore, 12,096 and 7,732 genes were negatively and positively correlated with *CXCL3* expression, respectively (Figure 9(c1)). Among them, 50 genes had a notable positive or negative correlation with *CXCL3* expression in COAD patients (Figures 9(c2) and 9(c3)). Expression of *CXCL3* was positively associated with the expression of *CXCL1* (PCO = 0.8921, *P* = 4.226*e*–132) (Figure 10(c1)), *CXCL2* (PCO = 0.8728, *P* = 1.601*e*–119) (Figure 10(c2)), and *ZC3H12A* (PCO = 0.6707, *P* = 7.446*e*–51) (Figure 10(c3)). Our results showed that 8,680 and 11,148 genes were negatively and positively correlated with *CXCL5* expression, respectively (Figure 9(d1)). Among them, 50 genes had a notable positive or negative correlation with *CXCL5* expression in COAD patients (Figures 9(d2) and 9(d3)). *CXCL5* expression was positively associated with the expression of *IL24* (PCO = 0.7438, *P* = 5.884*e*–68) (Figure 10(d1)), *IL8* (PCO = 0.7269, *P* = 1.632*e*–63) (Figure 10(d2)), and *MMP3* (PCO = 0.7213, *P* = 4.269*e*–62) (Figure 10(d3)). Our results suggested that 8,605 and 11,223 genes were negatively and positively correlated with *CXCL6* expression, respectively (Figure 9(e1)). Among them, 50 genes had a marked positive or negative correlation with *CXCL6* expression in COAD patients (Figures 9(e2) and 9(e3)). *CXCL6* expression was positively associated with the expression of *CXCL5* (PCO = 0.7105, *P* = 1.689*e*–59) (Figure 10(e1)), *MMP3* (PCO = 0.6904, *P* = 5.921*e*–55) (Figure 10(e2)), and *IL8* (PCO = 0.6833, *P* = 1.935*e*–53) (Figure 10(e3)). In addition, 9,079 and 10,749 genes were negatively and positively correlated with *CXCL8* expression, respectively (Figure 9(f1)). Among them, 50 genes had a significant positive or negative correlation with *CXCL8* expression in COAD patients (Figures 9(f2) and 9(f3)). *CXCL8* expression was positively associated with *GPR109B* (PCO = 0.7712, *P* = 5.939*e*–76) (Figure 10(f1)), *IL1B* (PCO = 0.7623, *P* = 3.25*e*–73) (Figure 10(f2)), and *OSM* (PCO = 0.7593, *P* = 2.368*e*–72) (Figure 10(f3)). Furthermore, 9,517 and 10,311 genes were negatively and positively correlated with *CXCL11* expression, respectively (Figure 9(g1)). Among them, 50 genes had a significant positive or negative correlation with *CXCL11* expression in COAD patients (Figures 9(g2) and 9(g3)). *CXCL11* expression was positively associated with *CXCL10* (PCO = 0.8389, *P* = 1.299*e*–101) (Figure 10(g1)), *UBD* (PCO = 0.7214, *P* = 3.935*e*–62) (Figure 10(g2)), and *IDO1* (PCO = 0.7116, *P* = 9.137*e*–60) (Figure 10(g3)). Moreover, 8,017 and 11,811 genes were negatively and positively correlated with *CXCL12* expression, respectively (Figure 9(h1)). Among them, 50 genes had a significant positive or negative correlation with *CXCL12* expression in COAD patients (Figures 9(h2) and 9(h3)). *CXCL12* expression was positively associated with *NPR1* (PCO = 0.804, *P* = 3.835*e*–87) (Figure 10(h1)), *SLIT3* (PCO = 0.8013, *P* = 3.915*e*–86) (Figure 10(h2)), and *SHE* (PCO = 0.7966, *P* = 1.928*e*–84) (Figure 10(h3)). Our results showed that 8,779 and 11,049 genes were negatively and positively correlated with *CXCL13* expression, respectively (Figure 9(i1)). Among them, 50 genes had a significant positive or negative correlation with *CXCL13* expression in COAD patients (Figures 9(i2) and 9(i3)). *CXCL13* expression was positively associated with expression of *TIGIT* (PCO = 0.8089, *P* = 5.598*e*–89) (Figure 10(i1)), *SH2D1A* (PCO = 0.7857, *P* = 1.229*e*–80) (Figure 10(i2)), and *SIRPG* (PCO = 0.7854, *P* = 1.508*e*–80) (Figure 10(i3)). In addition, 8,724 and 11,104 genes were negatively and positively correlated with *CXCL14* expression, respectively (Figure 9(j1)). Among them, 50 genes had a significant positive or negative correlation with *CXCL14* expression in COAD patients (Figures 9(j2) and 9(j3)). *CXCL14* expression was positively associated with the expression of *D4S234E* (PCO = 0.7057, *P* = 2.24*e*–58) (Figure 10(j1)), *TNFSF11* (PCO = 0.6172, *P* = 3.643*e*–41) (Figure 10(j2)), and *COL9A1* (PCO = 0.6154, *P* = 7.338*e*–41) (Figure 10(j3)). Furthermore, 9,737 and 10,091 genes were negatively and positively correlated with *CXCL16* expression, respectively (Figure 9(k1)). Among them, 50 genes had a significant positive or negative correlation with *CXCL16* expression in COAD patients (Figures 9(k2) and 9(k3)). *CXCL16* expression was positively associated with the expression of *ZMYND15* (PCO = 0.7944, *P* = 1.175*e*–83) (Figure 10(k1)), *FLII* (PCO = 0.6123, *P* = 2.248*e*–40) (Figure 10(k2)), and *NDEL1* (PCO = 0.6072, *P* = 1.486*e*–39) (Figure 10(k3)). We also found that 10,483 and 9,345 genes were negatively and positively correlated with *CXCL17* expression, respectively (Figure 9(l1)). Among them, 50 genes had a significant positive or negative correlation with *CXCL17* expression in COAD patients (Figures 9(l2) and 9(l3)). *CXCL17* expression was positively associated with the expression of *FAM83A* (PCO = 0.4586, *P* = 4.148*e*–21) (Figure 10(l1)), *GPR110* (PCO = 0.435, *P* = 6.333*e*–19) (Figure 10(l2)), and *SEMG1* (PCO = 0.402, *P* = 3.753*e*–16) (Figure 10(l3)). Finally, we found that 10,446 and 9,382 genes were negatively and positively correlated with *VEGFA* expression, respectively (Figure 9(m1)). Among them, 50 genes had a significant positive or negative correlation with *VEGFA* expression in COAD patients (Figures 9(m2) and 9(m3)). *VEGFA* expression was positively associated with the expression of *GTPBP2* (PCO = 0.5773, *P* = 4.639*e*–35) (Figure 10(m1)), *CCNL1* (PCO = 0.5422, *P* = 2.411*e*–30) (Figure 10(m2)), and *CREBZF* (PCO = 0.516, *P* = 3.606*e*–27) (Figure 10(m3)).

### 3.8. Immune Cell Infiltration and CXC Chemokine-VEGFA Network Expression

*CXCL1* expression in COAD patients was positively associated with CD8+ T cell infiltration, neutrophils, and dendritic cells (*P* < 0.05) (Figure 11(a)). However, macrophages were negatively associated with *CXCL1* expression (*P* < 0.01) (Figure 11(a)). In addition, neutrophil infiltration was positively associated with the expression of *CXCL2* and *CXCL3* (*P* < 0.001) (Figures 11(b) and 11(c)). However, macrophages were negatively associated with *CXCL2* and *CXCL3* expression (*P* < 0.001) (Figures 11(b) and 11(c)). Furthermore, expression levels of *CXCL5/6/8* in patients with COAD were positively associated with the infiltration of CD8+ T cells, macrophages, neutrophils, and dendritic cells (*P* < 0.01) (Figures 11(d)–11(f)). B cells, CD8+ T cells, CD4+ T cells, macrophages, neutrophils, and dendritic cells were positively associated with *CXCL11/12/13/16* expression (*P* < 0.01) (Figures 11(g)–11(i) and 11(k)). The expression level of *CXCL14* in patients with COAD was positively associated with the infiltration of CD8+ T cells, CD4+ T cells, neutrophils, and dendritic cells (*P* < 0.05) (Figure 11(j)). B cells were positively associated with *CXCL17* expression (*P* < 0.001) (Figure 11(l)). CD4+ T cells were positively associated with *VEGFA* expression (*P* < 0.01) (Figure 11(m)).

## 4. Discussion

Tumor angiogenesis plays a vital role in tumorigenesis, proliferation, and metastasis. In recent years, studies have identified *VEGFA* and CXC chemokines as important participants in angiogenesis, particularly tumor angiogenesis [14, 15, 26–28]. The expression levels of CXC chemokines and *VEGFA* have been studied in a range of tumor types; however, findings are contradictory with regard to colonic adenocarcinomas [29, 30]. This study investigated expression level, gene regulatory network, prognostic value, and target prediction of the CXC chemokine-VEGFA network for COAD from a tumor angiogenesis perspective.

In this study, we also examined the potential correlation between pathological stage and differential expression of COAD. The expression of *CXCL1/2/3/5/6/8/11/16/17* and *VEGFA* was upregulated in patients with COAD compared with that in individuals without COAD. Patients with COAD also showed downregulated *CXCL12/13/14* expression. The results were similar to those reported in a previous study in patients with COAD [30] and contradicted those reported previously in patients with colorectal cancer [29]. This may be due to the small sample size and the variable types of colorectal cancer. We further attempted to explain the different expression levels by investigating promoter methylation and gene alteration in patients with COAD, as these factors affect tumor cell proliferation, angiogenesis, and metastasis. We observed that patients with COAD had different rates of genetic alteration in their genes. Moreover, the promoter methylation levels of *CXCL5/6/12/14* and *VEGFA* were higher in patients with COAD than those in healthy individuals. Conversely, the promoter methylation levels of *CXCL1/2/3/11/13/17* were lower in patients with COAD. Thus, we hypothesized that genetic methylation and alteration within the CXC chemokine-VEGFA network might be the leading cause of abnormal gene expression levels in patients with COAD.

We also observed a notable correlation between the *CXCL9/10/11* and *VEGFA* expression and the pathological stage of COAD. Furthermore, the survival of patients with COAD was higher with low *VEGFA* or high *CXCL8/11/14* expression levels. Therefore, the expression levels of *CXCL8/11/14* and *VEGFA* may be potential prognostic indicators for COAD. *CXCL8/11/14* and VEGFA promote tumor angiogenesis in different ways [31–33]. Thus, they may affect the prognosis of patients with COAD through multiple biological functions.

The potential functions and interactions of the CXC chemokine-VEGFA network were further explored in this study. They were found to be complex and tightly connected. CXC chemokines and *VEGFA* may promote cancer progression, and this could be through a potential interaction network. Genes in the network were mainly involved in cytokine receptor binding, chemokine and cytokine activity, leukocyte chemotaxis, and migration, all of which are closely related to angiogenesis. For instance, IL-8 (*CXCL8*) promotes tumor angiogenesis by binding to CXCR1 and CXCR2 receptors [34]. In addition, increasing the antitumor activity of cytokine-induced killer cells could reduce tumor proliferation and angiogenesis [35]. Collectively, these results suggest that the CXC chemokine-VEGFA network may influence the development of COAD by increasing tumor angiogenesis.

Furthermore, the functions of the CXC chemokine-VEGFA network in patients with COAD were mainly related to chemokine activity, cytokine activity, and growth factor activity, as demonstrated by GO enrichment analysis, all of which are closely related to tumor angiogenesis. More studies are needed to confirm the mechanism by which this happens. In this study, we further found through KEGG pathway analysis that the cytokine–cytokine receptor interaction signaling pathway, IL-17 signaling pathway, and NF-*κ*B signaling pathway were highly involved in the CXC chemokine-VEGFA network in COAD patients, all of which are highly related to tumor angiogenesis [36, 37]. Therefore, the respective regulation of these pathways may serve as a potential treatment strategy for patients with COAD.

Mutated or altered transcription factors represent a unique class of drug targets that mediate aberrant gene expression, and the development of corresponding targeting drugs may impact future cancer treatments. Thus, the targets and regulators of the CXC chemokine-VEGFA network in COAD patients were further analyzed. The transcription factor targets of the CXC chemokine-VEGFA network in patients with COAD were identified. RELA, NFKB1, ZFP36, XBP1, HDAC2, SP1, ATF4, EP300, BRCA1, ESR1, HIF1A, EGR1, STAT3, and JUN were deemed crucial regulatory factors. Our results showed that these factors have potential functions in regulating tumor angiogenesis by targeting *VEGFA*. Studies have shown that RELA, NFKB1, HDAC2, SP1, ATF4, EP300, BRCA1, ESR1, HIF1A, EGR1, STAT3, and JUN regulate tumor angiogenesis, thus affecting tumor growth and prognosis [27, 28, 38–48]. However, the role of ZFP36 and XBP1 in tumor angiogenesis has not yet been reported. miRNAs also play a crucial role in regulating gene expression. miRNAs suppress target gene expression by targeting their 3′-untranslated regions. miRNA target discovery may ultimately help elucidate the underlying mechanisms of tumorigenesis. Thus, CXC chemokine-VEGFA network-associated miRNA targets in patients with COAD were further explored. Most miRNAs (miR-218, miR-493, miR-221, miR-222, miR-423, miR-378, miR-381, miR-210, miR-382, and miR-199A) have been shown to regulate tumor angiogenesis [49–52]. In summary, our study provides the basis for potential therapeutic strategies for treating COAD by predicting regulated factors and miRNA targets. This study had limitations; no cell line in vitro or in vivo studies were performed to further validate our results.

The correlation between CXC chemokine-VEGFA network expression and differentially expressed genes in COAD patients was explored in this study. We found that in patients with COAD, approximately 20,000 genes were negatively or positively correlated with CXC chemokine-VEGFA network expression. From these, we screened for genes with the highest correlation with CXC chemokines and *VEGFA*. Some of the genes with the highest correlation (*ZC3H12A,* IL24, *MMP3*, *IL1B*, *OSM*, *IDO1*, *NPR1*, and *TIGIT*) were positively associated with tumor angiogenesis [53, 54]. Regulation of these cancer-related genes may offer an alternative therapeutic strategy for the treatment of patients with COAD. Immune infiltration is highly related to the clinical prognosis of tumors. Immune cells reach the tumor site through vascular transport, and vascularization of tumors is a process mediated by angiogenesis. We observed that CXC chemokine-VEGFA network expression, which regulates angiogenesis, is correlated with the infiltration of immune cells. This infiltration involved CD4+ T cells, CD8+ T cells, neutrophils, macrophages, and dendritic cells. Improving immune cell infiltration in COAD by developing drugs that act on the CXC chemokine-VEGFA network or CXC chemokines and *VEGFA*-related regulatory targets may serve as a viable therapeutic oncology approach.

## 5. Conclusions

In this study, we determined the expression levels and gene regulatory network of the CXC chemokine-VEGFA network, which plays a vital role in angiogenesis in COAD. We also identified new prognostic biomarkers and therapeutic targets. These findings provide insight into the study and treatment of COAD.

## Figures and Tables

**Figure 1:** The transcription of CXC chemokine-*VEGFA* network in COAD (UALCAN). (a1–m1) The transcription expression of *CXCL1/2/3/5/6/8/11/12/13/14/16/17* and *VEGFA* in COAD based on sample types. (a2–m2) The transcription expression of *CXCL1/2/3/5/6/8/11/12/13/14/16/17* and *VEGFA* in COAD based on the sex of the patient. (a3–m3) The transcription expression of *CXCL1/2/3/5/6/8/11/12/13/14/16/17* and *VEGFA* in COAD based on individual cancer stages. Sample type denotes normal and patient groups. Gender denotes male and female. A Student's *t*-test was used for the comparative analysis, ^∗^*P* < 0.05; ^∗∗^*P* < 0.01; ^∗∗∗^*P* < 0.001.

**Figure 2:** The protein expression of CXC chemokine-*VEGFA* network in COAD (Human Protein Atlas). (a1–h1) The protein expression of *CXCL5/8/11/12/13/14/16* and *VEGFA* in normal colon tissue, respectively. (a2–h2) The protein expression of *CXCL5/8/11/12/13/14/16* and *VEGFA* in COAD tissue, respectively. Note: the Human Protein Atlas database does not include immunohistochemical data for CXCL1/2/3/6/17 in COAD tissue.

**Figure 3:** Correlation between the pathological stage and different expressed CXC chemokine-*VEGFA* network of COAD patients (GEPIA): (a) *CXCL9*; (b) *CXCL10*; (c) *CXCL11*; (d) *VEGFA*. Notably, our results did not show statistically significant data. A Student's *t*-test was used for the comparative analysis.

**Figure 4:** The prognostic value of CXC chemokine-*VEGFA* network in COAD (GEPIA). The overall survival curve of (a) *CXCL8* and (b) *CXCL14*. The disease-free survival of (c) *CXCL11* and (d) *VEGFA*. Note: our results did not show statistically significant data.

**Figure 5:** Genetic alteration of CXC chemokine-*VEGFA* network in COAD (cBioPortal).

**Figure 6:** Promoter methylation of CXC chemokine-*VEGFA* network in COAD (UALCAN). (a) The promoter methylation level of *CXCL1* in healthy individuals and COAD patients. (b) The promoter methylation level of *CXCL2* in healthy individuals and COAD patients. (c) The promoter methylation level of *CXCL3* in healthy individuals and COAD patients. (d) The promoter methylation level of *CXCL5* in healthy individuals and COAD patients. (e) The promoter methylation level of *CXCL6* in healthy individuals and COAD patients. (f) The promoter methylation level of *CXCL11* in healthy individuals and COAD patients. (g) The promoter methylation level of *CXCL12* in healthy individuals and COAD patients. (h) The promoter methylation level of *CXCL13* in healthy individuals and COAD patients. (i) The promoter methylation level of *CXCL14* in healthy individuals and COAD patients. (j) The promoter methylation level of *CXCL17* in healthy individuals and COAD patients. (k) The promoter methylation level of *VEGFA* in healthy individuals and COAD patients. Note: our results did not show statistically significant data. A Student's *t*-test was used for the comparative analysis, ^∗^*P* < 0.05; ^∗∗^*P* < 0.01; ^∗∗∗^*P* < 0.001.

**Figure 7:** Interaction analyses of CXC chemokine-*VEGFA* network in COAD. (a) PPI network of CXC chemokine-*VEGFA* network in COAD (STRING). (b) Network and function analyses of CXC chemokine-*VEGFA* network in COAD (GeneMANIA).

**Figure 8:** GO function and KEGG pathway enrichment analyses of CXC chemokine-*VEGFA* network in COAD (Metascape). (a) Biological processes in COAD. (b) Molecular functions in COAD. (c) KEGG pathway analysis in COAD.

**Figure 9:** Genes differentially expressed in correlation with CXC chemokine-*VEGFA* network in COAD (LinkedOmics). (a1–m1) Pearson's correlation test was used to analyze correlations between *CXCL1/2/3/5/6/8/11/12/13/14/16/17*, *VEGFA*, and genes differentially expressed in COAD, respectively. (a2–m2, a3–m3) Heat maps showing genes positively and negatively correlated with *CXCL1/2/3/5/6/8/11/12/13/14/16/17* and *VEGFA* in COAD, respectively (top 50 genes).

**Figure 10:** Gene expression correlation analysis of CXC chemokine-*VEGFA* network in COAD (LinkedOmics). The scatter plot shows Pearson's correlation of *CXCL1* expression with expression of (a1) *CXCL3*, (a2) *CXCL2*, and (a3) *ZC3H12A* in COAD; Pearson's correlation of *CXCL2* expression with expression of (b1) *CXCL3*, (a2) *CXCL1*, and (b2) *ZC3H12A* in COAD; Pearson's correlation of *CXCL3* expression with expression of (a1) *CXCL1*, (b1) *CXCL2*, and (b3) *ZC3H12A* in COAD; Pearson's correlation of *CXCL5* expression with expression of (c1) *IL24*, (c2) *IL8*, and (c3) *MMP3* in COAD; Pearson's correlation of *CXCL6* expression with expression of (d1) *CXCL5*, (d2) *MMP3*, and (d3) *IL8* in COAD; Pearson's correlation of *CXCL8* expression with expression of (e1) *GPR109B*, (e2) *IL1B*, and (e3) *OSM* in COAD; Pearson's correlation of *CXCL11* expression with expression of (f1) *CXCL10*, (f2) *UBD*, and (f3) *IDO1* in COAD; Pearson's correlation of *CXCL12* expression with expression of (g1) *NPR1*, (g2) *SLIT3*, and (g3) *SHE* in COAD; Pearson's correlation of *CXCL13* expression with expression of (h1) *TIGIT*, (h2) *SH2D1A*, and (h3) *SIRPG* in COAD; Pearson's correlation of *CXCL14* expression with expression of (i1) *D4S234E*, (i2) *TNFSF11*, and (i3) *COL9A1* in COAD; Pearson's correlation of *CXCL16* expression with expression of (j1) *ZMYND15*, (j2) *FLII*, and (j3) *NDEL1* in COAD; Pearson's correlation of *CXCL17* expression with expression of (k1) *FAM83A*, (k2) *GPR110*, and (k3) *SEMG1* in COAD; and Pearson's correlation of *VEGFA* expression with expression of (l1) *GTPBP2*, (l2) *CCNL1*, and (l3) *CREBZF* in COAD.

**Figure 11:** The correlation between CXC chemokine-*VEGFA* network and immune cell infiltration in COAD (TIMER): (a) *CXCL1*; (b) *CXCL2*; (c) *CXCL3*; (d) *CXCL5*; (e) *CXCL6*; (f) *CXCL8*; (g) *CXCL11*; (h) *CXCL12*; (i) *CXCL13*; (j) *CXCL14*; (k) *CXCL16*; (l) *CXCL17*; (m) *VEGFA*.

**Table 1:** Key regulated factor of CXCL and *VEGFA* in COAD (TRRUST).

Key TF	Description	Regulated gene	*P* value	FDR
RELA	v-rel reticuloendotheliosis viral oncogene homolog A (avian)	CXCL1, CXCL2, CXCL5, CXCL8, CXCL12, VEGFA	2.44*e* − 08	1.78*e* − 07
NFKB1	Nuclear factor of kappa light polypeptide gene enhancer in B cells 1	CXCL1, CXCL2, CXCL5, CXCL8, CXCL12, VEGFA	2.54*e* − 08	11.78*e* − 07
ZFP36	ZFP36 ring finger protein	CXCL8, VEGFA	1.22*e* − 05	5.71*e* − 05
XBP1	X-box-binding protein 1	CXCL8, VEGFA	7.44*e* − 05	0.000261
HDAC2	Histone deacetylase 2	CXCL8, VEGFA	0.000152	0.000426
SP1	Sp1 transcription factor	CXCL1, CXCL5, CXCL14, VEGFA	0.000231	0.000515
ATF4	Activating transcription factor 4 (tax-responsive enhancer element B67)	CXCL8, VEGFA	0.000257	0.000515
EP300	E1A-binding protein p300	CXCL8, VEGFA	0.000661	0.00106
BRCA1	Breast cancer 1, early onset	CXCL1, VEGFA	0.000685	0.00106
ESR1	Estrogen receptor 1	CXCL12, VEGFA	0.00121	0.0017
HIF1A	Hypoxia inducible factor 1, alpha subunit (basic helix-loop-helix transcription factor)	CXCL12, VEGFA	0.00144	0.00184
EGR1	Early growth response 1	CXCL8, VEGFA	0.00162	0.00189
STAT3	Signal transducer and activator of transcription 3 (acute-phase response factor)	CXCL8, VEGFA	0.00415	0.00447
JUN	Jun proto-oncogene	CXCL8, VEGFA	0.00456	0.00456

**Table 2:** The miRNA target of CXCL and *VEGFA* in COAD (LinkedOmics).

Cancer type	Gene	Gene set	Leading edge number	*P* value	FDR
COAD	CXCL1	TCCAGAG, MIR-518C	47	0.001	0.013584
		GTATTAT, MIR-369-3P	86	0.001	0.018113
		ATATGCA, MIR-448	64	0.001	0.024150
	CXCL2	TCCAGAG, MIR-518C	51	0.001	0
		AAGCACA, MIR-218	143	0.001	0
		ATGTACA, MIR-493	130	0.001	0
	CXCL3	ATATGCA, MIR-448	92	0.001	0
		GTATTAT, MIR-369-3P	100	0.001	0
		ATGTAGC, MIR-221, MIR-222	49	0.001	0.00052445
	CXCL13	ACCGAGC, MIR-423	3	0.015625	0.028853
	CXCL14	GTCAGGA, MIR-378	18	0.0051151	0.02937
		CTTGTAT, MIR-381	55	0.001	0.031719
		ACGCACA, MIR-210	3	0.0031348	0.037446
	CXCL17	GTATTAT, MIR-369-3P	97	0.001	0.0039402
		ACAACTT, MIR-382	18	0.001	0.023641
		CGTCTTA, MIR-208	5	0.001	0.029552
	VEGFA	GTACAGG, MIR-486	16	0.0030120	0.053189
		CTACTGT, MIR-199A	52	0.001	0.054125

## Data Availability

The UALCAN (http://ualcan.path.uab.edu/analysis.html), Human Protein Atlas (https://www.proteinatlas.org/), GEPIA (http://gepia.cancer-pku.cn/index.html), cBioPortal (http://cbioportal.org), STRING (https://string-db.org/cgi/input.pl), GeneMANIA (http://www.genemania.org), Metascape (https://metascape.org), TRRUST (https://www.grnpedia.org/trrust/), LinkedOmics (http://www.linkedomics.org/), and TIMER (https://cistrome.shinyapps.io/timer/) were used.

## Abbreviations

COAD: Colon adenocarcinoma
VEGFA: Vascular endothelial growth factor A
GEPIA: Gene expression profiling analysis
GO: Gene Ontology
KEGG: Kyoto Encyclopedia of Genes and Genomes
TCGA: The Cancer Genome Atlas
RELA: v-rel reticuloendotheliosis viral oncogene homolog A
NFKB1: Nuclear factor of kappa light polypeptide gene enhancer in B cells 1
ZFP36: ZFP36 ring finger protein
XBP1: X-box-binding protein 1
HDAC2: Histone deacetylase 2
ATF4: Activating transcription factor 4
EP300: E1A-binding protein p300
EGR1: Early growth response 1
STAT3: Signal transducer and activator of transcription 3
JUN: Jun proto-oncogene
SP1: Sp1 transcription factor
BRCA1: Breast cancer 1
ESR1: Estrogen receptor 1
HIF1A: Hypoxia inducible factor 1 alpha subunit.
